The article "Application of Preoperative Adductor Canal Block Coupled with General Anaesthesia in Elderly Patients Undergoing Total Knee Arthroplasty" was retracted in 2023. Reasons: unreliable results or conclusions; lack of ethics approval or compliance; concerns about the data; concerns about the peer review.

# Application of Preoperative Adductor Canal Block Coupled with General Anaesthesia in Elderly Patients Undergoing Total Knee Arthroplasty

**DOI:** 10.1155/2022/3071665

**Published:** 2022-10-13

**Authors:** Haiyan Huang, A-feng Zhang, Huaixin Gao, Na Li, Minggang Fang

**Affiliations:** ^1^Anesthesiology Department, Nuclear Industry 215 Hospital of Shaanxi Province, Shaanxi 712000, China; ^2^Anesthesiology Department, Xianyang Central Hospital, Xianyang, Shaanxi Province, China

## Abstract

**Objective:**

To investigate the clinical application of preoperative adductor canal block combined with general anaesthesia in elderly patients with total knee arthroplasty.

**Methods:**

Seventy-four patients scheduled for elective TKA in Shaanxi Nuclear Industry Hospital No. 215 were selected and were assigned into group A (continuous ACB prior to the induction of anaesthesia) and group B (continuous ACB after extraction of the tracheal catheter post-operatively) according to the random number table method. Pre and postoperative plasma adrenaline and noradrenaline levels were measured; mean arterial pressure (MAP) and heart rate (HR) were recorded at the admission and the surgical skin incision; intraoperative sufentanil dosage, number of analgesic pump presses at 48 h postoperatively; postoperative adverse effects and length of stay were recorded; resting and active VAS pain scores were assessed at 4, 8, 12, 24, and 48 h postoperatively.

**Results:**

Group B experienced a substantial increase in MAP and HR at the time of surgical skin incision, while group A registered a smaller change and a stable haemodynamic profile (*P* < 0.05). The plasma adrenaline and norepinephrine concentrations in group B were elevated compared to the preoperative period, differentially with group A. Group A received less intraoperative sufentanil than Group B (*P* < 0.05).

**Conclusion:**

Collectively, postoperative resting VAS scores and active VAS scores remained lower in TKA patients who were subjected to preoperative and postoperative ACB, while preoperative ACB in conjunction with general anaesthesia decreased intraoperative sufentanil dosage, contained the surgical stress response, and maintained a stable intraoperative haemodynamic state, in what is probably a preferable option for elderly patients undergoing TKA. This study has served as a reference for postoperative patients to reduce their medication and for clinicians in the treatment going forward.

## 1. Introduction

Total knee arthroplasty (TKA) is universally acclaimed as an efficacious treatment for severe degenerative knee changes, delivering substantial improvements in knee function and quality of life for patients [1]. Approximately 15% of females and 6% of males in the Asian elderly population over 60 years suffer from osteoarthritis of the knee. The majority of patients eventually opt for TKA for treatment. Notwithstanding considerable advances in surgical technique or prosthesis design, acute postoperative pain among TKA patients remains in the forefront of clinicians' minds as one of the most pressing issues to be addressed. Acute postoperative pain impairs not only early activities and functional exercise but also carries an increased risk of postoperative knee stiffness and deep vein thrombosis [2]. Almost 60% of patients experienced moderate to severe pain following total knee arthroplasty, and 25% of these patients may even develop relevant complications such as prolonged hospital stays, unplanned hospitalisations, and readmissions. The early initiation of functional exercise for improved postoperative recovery necessitates adequate management for postoperative pain.

The article "Application of Preoperative Adductor Canal Block Coupled with General Anaesthesia in Elderly Patients Undergoing Total Knee Arthroplasty" was retracted in 2023. Reasons: unreliable results or conclusions; lack of ethics approval or compliance; concerns about the data; concerns about the peer review.

Conventional intravenous, oral, and intramuscular analgesic drugs can alleviate soreness with unsatisfactory outcomes [3]. Epidural analgesia is highly effective and available for postoperative management of acute pain, but indwelling epidural catheters entail risks of infection and bleeding as well as complications such as urinary retention and hypotension [4]. Perioperative multimodal analgesia, mainly peripheral nerve block, is currently advocated for postoperative analgesia after TKA [5]. Peripheral nerve blocks, including the adductor canal block (ACB) and femoral nerve block (FNB), are broadly accepted as part of a multimodal pain relief protocol in patients undergoing total knee arthroplasty owing to their effectiveness in reducing postoperative opioid application and preserving lower limb motion. Nonetheless, the analgesic coverage of ACB is confined to the anteromedial portion of the knee joint. Therefore, many investigators have reported better analgesic efficacy using peripheral nerve blocks combined with periarticular injections (PAI) during TKA. Compared to FNB, ACB is the most extensively embraced ultrasound-guided block for preserving motion. ACB is deemed to block the posterior branches of the saphenous, medial femoral and foraminal nerves (approximately 8% of the motor block) while retaining quadriceps strength better than FNB [6].

Over the recent years, ultrasound guidance enhances the success rate of ACB and has gained extensive acceptance as a technique to control pain in the aftermath of TKA. However, no researcher has proposed if there is an ideal time to utilize ACB for maximum benefit. The objective of this study was therefore to investigate the effect of ACB on the effectiveness of anaesthesia, quadriceps muscle strength, and postoperative inflammatory response in patients undergoing knee arthroscopy. Preoperative ultrasound-guided continuous ACB coupled with general anaesthesia was used in this study for TKA in older patients, with superior and satisfactory outcomes, as stated.

The article "Application of Preoperative Adductor Canal Block Coupled with General Anaesthesia in Elderly Patients Undergoing Total Knee Arthroplasty" was retracted in 2023. Reasons: unreliable results or conclusions; lack of ethics approval or compliance; concerns about the data; concerns about the peer review.

## 2. Materials and Methods

### 2.1. General Data

We chose a clinical trial that had undergone prospective merit review, whose version of the study protocol submitted to the IRB was available, and that was currently underway. Patients scheduled for elective TKA in our hospital from December 2020 to December 2021 were selected, regardless of gender, aged 65-82 years old, weighing 55-82 kg, with ASA class II or III. Participants were allocated in a 1: 1 ratio to 1 of the 2 groups. Patients were randomly assigned to groups by means of a password-protected web-based system developed and maintained by Exeter Clinical Trials Unit. Allocation was stratified by centre and minimised on patient age, sex, and presence of FBSS. Once the patient completed the screening interview and baseline data collection interview, the researcher accessed the randomisation website using a unique username and password.

#### 2.1.1. Ethical Considerations

This study is an RCT which unmasked the two treatment allocation. The study adheres to the tenets of The Declaration of Helsinki and is registered at http://www.controlled-trials.com/ (trial registration number: ISRCT728038223). Ethical approval was granted by the Ethics Committee. The trial is monitored by a Trial Management Group, a Trial Steering Committee, and a Data and Safety Monitoring Committee.

#### 2.1.2. Inclusion and Exclusion Criteria

Inclusion criteria: (1) patients undergoing unilateral TKA; (2) patients who required for postoperative analgesia; (3) patients who voluntarily participated in this study. Exclusion criteria: (1) patients with a history of central nervous system disease; (2) patients receiving long-term opioid analgesics; (3) patients with infection of the skin at the puncture site or route; and (4) patients with abnormal coagulation function and obvious abnormalities in heart, lung, liver, and kidney function.

### 2.2. Anaesthesia Methods

All patients were given intravenously 0.05 mg/kg midazolam (Jiangsu Enhua Pharmaceutical Co., Ltd., Lot No. MD201105), 0.3 mg/kg etomidate (Jiangsu Enhua Pharmaceutical Co., Ltd., Lot No. YT201026), 0.3-0.5 *μ*g/kg sufentanil (Yichang Renfu Pharmaceutical Co., Ltd., GuoYaoZhunZi H20054171), and 1.0 mg/kg rocuronium bromide (Zhejiang Xianju Pharmaceutical Co., Ltd., GuoYaoZhunZi H20123188) for the induction of general anaesthesia. Following tracheal intubation, mechanical ventilation was performed with a tidal volume of 6-8 mL/kg at a frequency of 12 times/min, with PaCO_2_ maintained at 35-45 mmHg. The depth of anaesthesia was sustained intraoperatively with rocuronium bromide, sufentanil, and propofol (Xi'an Lipan Pharmaceutical Co., Ltd., GuoYaoZhunZi 20163040), and the EEG bispectral index (BIS) score was recorded in the range of 40-60.

The article "Application of Preoperative Adductor Canal Block Coupled with General Anaesthesia in Elderly Patients Undergoing Total Knee Arthroplasty" was retracted in 2023. Reasons: unreliable results or conclusions; lack of ethics approval or compliance; concerns about the data; concerns about the peer review.

### 2.3. Grouping and Treatment

Seventy-two patients were assigned into group A (continuous ACB prior to the induction of anaesthesia) and group B (continuous ACB after extraction of the tracheal catheter postoperatively) according to the random number table method. The nerve blocking was performed by the same senior anaesthetist, with a portable ultrasonic instrument and a continuous plexus block kit (Contiplex D, B. Braun Melsungen AG, Germany) used in both groups as follows. The patient is placed in a supine position with the legs slightly apart, and the affected limb slightly abducted and externally rotated. A high-frequency ultrasound probe is placed across the medial thigh, perpendicular to the femur, and the short-axis section of the thigh is scanned. The suture, longissimus, and medial femoral muscles are identified in the ultrasound image. Using an in-plane technique, the tip of the nerve block needle is placed through the suture muscle to a position between the femoral artery and the saphenous nerve, and 20 ml of 0.25% ropivacaine is injected after confirming the position.

The perineural interspace was widened after injection of a loading dose of local anaesthetic in both groups; the, the needle tip was adjusted to the appropriate position, and the indwelling catheter was inserted along the puncture needle into the perineural area; the indwelling catheter was withdrawn from the puncture needle at a depth of 6 cm, secured with proper sutures, and the catheter was fixed with a sterile film dressing and connected to a postoperative self-administered analgesia pump before being sent back to the ward. The analgesic drug used was 0.25% ropivacaine (250 ml), with a PCA dose of 5 ml, a locking time to be set at 30 min and an infusion rate of 5 ml/h for 48 h.

### 2.4. Observation Indicators

The MAP and HR were recorded at the time of admission and surgical skin incision. 3-5 mL of venous blood was collected from the forearm on the noninfused side at the time of admission and at the end of surgery, and the plasma epinephrine and norepinephrine levels were measured using a modified fluorometric method after separation and extraction of serum. Intraoperative sufentanil dosage, number of analgesic pump presses at 48 h postoperatively; postoperative adverse effects and comparative length of stay were recorded; resting and active VAS pain scores at 4, 8, 12, 24, and 48 h postoperatively were assessed using a visual analogue scale (VAS score ranging 0-10, with 0 indicating no pain, and 10 indicating intolerable severe pain).

The article "Application of Preoperative Adductor Canal Block Coupled with General Anaesthesia in Elderly Patients Undergoing Total Knee Arthroplasty" was retracted in 2023. Reasons: unreliable results or conclusions; lack of ethics approval or compliance; concerns about the data; concerns about the peer review.

### 2.5. Statistical Methods

The sample size was calculated by using Gpower® (V3.1.9.2 standard version) based on the scores of intraoperative sufentanil dosage of the first 5 patients in each group of the pretest. A statistical efficiency of 1 − *β* = 0.9, a test criterion of *α* = 0.05, and a test efficacy of 90% were set from the preliminary pretest analysis, and 32 patients per group were calculated to be required. With an assumed lost-to-review rate of 15%, 74 patients were eventually recruited.

SPSS 18.0 software was adopted for statistical analysis. Continuous data were expressed as *x* ± *s*, and categorical data were presented as *n*/%. The Kolmogorov-Smirnov normality test was performed on the continuous observed indicator variables: Student's *t* test was conducted for the intergroup comparison as a normal distribution was conformed; otherwise, Mann–Whitney *U* test was performed. Categorical data were compared using the *χ*^2^ test or Fischer's exact test. *P* < 0.05 is defined as a statistically significant difference.

## 3. Results

One case in group A was withdrawn as the procedure was altered, and two cases in group B were excluded as the catheter for the continuous plexus block was dislodged; hence, the ultimate number of cases in groups A and B was 36 and 35, respectively. No significant differences were detected in gender, age, weight, and ASA grade across the two groups (Table 1).

### 3.1. Intergroup Comparison of MAP and HR at the Admission and at the Surgical Skin Incision

The intergroup comparison exhibited no difference in the MAP and HR on admission (*P* > 0.05). Group B experienced a substantial increase in MAP and HR at the time of surgical skin incision, while group A registered a smaller change and a stable haemodynamic profile (*P* < 0.05).  Table 2.

### 3.2. Intergroup Comparison of Plasma Adrenaline and Norepinephrine Content at Different Times

No difference was found in preoperative plasma epinephrine and norepinephrine levels across the two groups (*P* > 0.05). Postoperatively, groups B experienced a marked increase in plasma epinephrine and norepinephrine levels compared to group A (*P* < 0.05), Table 3.

### 3.3. Intergroup Comparison of Intraoperative Sufentanil Dosage, Frequency of Analgesic Pumps within 48 Hours, Adverse Postoperative Reactions, and Length of Hospital Stay

Intraoperative sufentanil dosage was inferior in group A than in group B, with statistically significant difference (*P* < 0.05). No statistically significant differences were found in the intergroup comparison in terms of the number of postoperative analgesic pump presses, postoperative adverse reaction, and length of hospital stay (*P* > 0.05). See Table 4.

The article "Application of Preoperative Adductor Canal Block Coupled with General Anaesthesia in Elderly Patients Undergoing Total Knee Arthroplasty" was retracted in 2023. Reasons: unreliable results or conclusions; lack of ethics approval or compliance; concerns about the data; concerns about the peer review.

### 3.4. Intergroup Comparison of VAS Scores at Resting State and Active State 4, 8, 12, 24, and 48 Hours Postoperatively

The intergroup comparison revealed no statistically significant difference with regard to VAS scores at rest and in the active state 4 to 48 hours postoperatively (*P* > 0.05).  Table 5.

## 4. Discussion

TKA is frequently adopted in the clinical management of advanced knee disease; to date, however, on account of the extensive intraoperative osteotomy and the large surgical incision, most patients may suffer from severe pain postoperatively [7]. Adequate postoperative analgesia alleviates pain symptoms and facilitates timely postoperative functional exercise in such patients, contributing to the early recovery of joint function [8]. Traditional epidural anaesthesia in elderly patients is characterised by reduced autonomic reflex strength and response rate, unstable blood pressure control, and inability to effectively maintain haemodynamic stability, thus rendering poorly tolerated anaesthesia. In addition, there is a high risk of epidural anaesthesia causing blockage of the nerves innervating the bladder sphincter, making it difficult for patients to urinate and retain urine after anaesthesia. It is a prevailing trend to use multimodal analgesia in the perioperative period, in which peripheral nerve blocks take on an influential role. In recent years, ultrasound-guided ACB has been widely accepted in the treatment of postoperative pain following TKA, and ACB can expedite the recovery of postoperative motor function after TKA [9, 10]. Multimodal analgesic modalities fully illustrate the benefits of ACB and reduce the adverse reactions and complications pertaining to postoperative analgesia [11]. Yet, how to exploit the maximum benefits of ACB has been sidelined. Therefore, the objective of this study was to assess the influence of ACB on reducing pain after TKA and to elucidate the optimal timing of ACB for better outcomes.

Intraoperative smooth haemodynamics, by which the risk of perioperative cardiovascular disease can be effectively reduced, is also the most essential requirement for anaesthesia, especially in elderly patients with impaired cardiovascular function [12]. The extent to which anaesthesia suppresses surgical stimulation is reflected on cardiovascular response, with blood pressure and HR being among the frequently cited indicators. The present study has demonstrated that the intraoperative dose of sufentanil in group A was less than that in group B, pointing to the effectiveness of preoperative ACB in suppressing intraoperative surgical stimulation. Group B experienced a substantial increase in MAP and HR at the time of surgical skin incision, while group A registered a smaller change and a stable haemodynamic profile. The stress response refers to a normal physiological phenomenon in surgical anaesthesia, a nonspecific defence response stimulated by a variety of factors in the perioperative period, but an above-normal or prolonged stress response activates the hypothalamic-pituitary-adrenocortical system, triggering an increase in the secretion of catecholamines, involving adrenaline and noradrenaline [13]. The findings of this study disclosed that the plasma adrenaline and norepinephrine concentrations in group B were elevated compared to the preoperative period, differentially with group A, which indicated that group A exhibited a milder stress response. Taken together, it has implied that preoperative ACB coupled with general anaesthesia could effectively reduce the stress response generated by surgery and maintain the intraorganic environment [14, 15].

The article "Application of Preoperative Adductor Canal Block Coupled with General Anaesthesia in Elderly Patients Undergoing Total Knee Arthroplasty" was retracted in 2023. Reasons: unreliable results or conclusions; lack of ethics approval or compliance; concerns about the data; concerns about the peer review.

In this study, no comparison of the use of other intraoperative anaesthetics was conducted to confirm alternative approaches to the suppression of surgical stress with anaesthesia. Virtually all patients in this study were given general anaesthesia under BIS guidance, and BIS scores were maintained in the range of 40-60 to ensure adequate depth of anaesthesia [16, 17]. Intraoperatively, group A required less sufentanil in comparison to group B, yet this difference was not remarkable, which may be indicative that even preoperative ACB may be required for opioid suppression of the injurious irritation associated with extensive osteotomy during TKA and the larger surgical incision, as ACB alone is less likelihood of conferring a complete knee pain block, primarily as the posterior and lateral parts of the knee would not be effectively blocked by ACB [18]. In addition, FNB is associated with a serious adverse effect of quadriceps weakness, which interferes with postoperative rehabilitation exercises and ambulation in TKA patients, thereby inducing serious complications such as lower limb venous thrombosis and falls. The ACB is assumed to serve the purpose of preserving quadriceps muscle strength since the block is performed distal to the motor fibre branches of the femoral nerve (with the exception of the nerve to the medial femoral muscle). Such is a point for clinicians to be aware of as well [19, 20].

On the subject of postoperative analgesia, both group A and B maintained low resting and active VAS scores from 4 to 48 hours postoperatively, endorsing the effectiveness of ACB in reducing acute postoperative pain after TKA [21]. It is universally appreciated that ACB is an ideal option for postoperative analgesia in TKA as it delivers a wider range of sensory blockade after TKA and exerts its analgesic effect without compromising quadriceps muscle strength [22, 23]. The reason lies in the fact that early postoperative walking with the knee in the extended position does not require much muscle strength in the quadriceps. Despite concerns that FNB may increase the risk of falls, no falls were observed in the patients in this study [24, 25].

The article "Application of Preoperative Adductor Canal Block Coupled with General Anaesthesia in Elderly Patients Undergoing Total Knee Arthroplasty" was retracted in 2023. Reasons: unreliable results or conclusions; lack of ethics approval or compliance; concerns about the data; concerns about the peer review.

This study differentiates from the traditional application of anaesthesia by using a peripheral nerve block to provide adequate control of postoperative pain. In this study, we investigated how the use of ACB during TKA works and provided some insight into the treatment and diagnosis of patients with degenerative knee disease. However, this study did not identify biomarkers of effectiveness or the mechanism on which the ACB used in this study was based for treatment. It is a direction for our future research. Some limitations abound in our study. Foremost, in this study, postoperative quadriceps muscle strength as well as knee mobility were not evaluated to further elaborate the impact of ACB on postoperative knee function recovery while attenuating acute postoperative pain. Secondly, this study was a single-centre study with a small sample size, and a larger sample size remains warranted for subsequent studies to confirm the superiority of preoperative ACB. Furthermore, the study was carried out in a centre where the procedure was performed by a number of different surgeons. Potential risks associated with the use of ACB are also identified, including the risk of muscle damage, neuropathy, and infection.

Collectively, postoperative resting VAS scores and active VAS scores remained lower in TKA patients who were subjected to preoperative and postoperative ACB, while preoperative ACB in conjunction with general anaesthesia decreased intraoperative sufentanil dosage, contained the surgical stress response, and maintained a stable intraoperative haemodynamic state, in what is probably a preferable option for elderly patients undergoing TKA. However, some limitations exist in this study and need to be analysed by clinicians in their specific choice of treatment. When conditions permit, an in vitro and in vivo trial will be conducted to investigate how ACB can improve symptoms after TKA.

## Figures and Tables

**Table 1:** Intergroup comparison of the general data.

Group	*n*	Gender (male/female)	Age (year old)	Weight (kg)	ASA (*n*)	
					II	III
A	36	20/16	72.83 ± 4.69	69.29 ± 7.93	22	14
B	35	18/17	72.44 ± 4.66	69.85 ± 7.54	23	12
*χ* ^2^/*t*		0.122	0.390	-0.308	0.162	
*P*		0.727	0.698	0.759	0.687	

The article "Application of Preoperative Adductor Canal Block Coupled with General Anaesthesia in Elderly Patients Undergoing Total Knee Arthroplasty" was retracted in 2023. Reasons: unreliable results or conclusions; lack of ethics approval or compliance; concerns about the data; concerns about the peer review.

**Table 2:** Intergroup comparison of MAP and HR at the admission and at the surgical skin incision ($\bar{x}\pm s$).

Group	*n*	MAP (mmHg)		HR (beats/min)	
		At the admission	Surgical skin incision	At the admission	Surgical skin incision
A	36	88.75±	87.61±	85.02±	83.18±
B	35	88.08±	93.42±	86.11±	88.45±
*t*		0.686	-5.923	-0.54	-3.512
*P*		0.495	0.001	0.591	0.001

**Table 3:** Intergroup comparison of plasma adrenaline and norepinephrine ($\bar{x}\pm s$).

Group	n	Adrenaline (ng/L)		Norepinephrine (ng/L)	
		Preoperation	Postoperation	Preoperation	Postoperation
A	36	33.1 ± 3.4	33.3 ± 5.5	152.1 ± 42.5	154.7 ± 47.8
B	35	32.7 ± 3.2	52.6 ± 8.4	151.4 ± 43.6	185.4 ± 49.6
*t*		0.239	36.571	0.334	17.615
*P*		0.217	0.001	0.167	0.001

**Table 4:** Intergroup comparison of intraoperative sufentanil dosage, frequency of analgesic pumps, adverse postoperative reactions, and length of hospital stay ($\bar{x}\pm s$, *n*/%).

Group	*n*	Sufentanil dosage (g)	Frequency of presses (times)	Adverse reactions (*n*/%)		Length of hospital stay (day)
				Nausea and vomiting	Cognitive dysfunction	
A	36	25.44 ± 5.9	13.2 ± 4.2	2 (5.5)	1 (2.7)	9.1 ± 1.5
B	35	38.8 ± 5.7	13.4 ± 4.3	1 (2.7)	0 (0.0)	8.9 ± 1.8
*χ* ^2^/*t*		-9.661	-0.174	3.247	1.267	0.142
*P*		0.000	0.862	0.354	1.000	0.888

**Table 5:** Intergroup comparison of postoperative VAS scores ($\bar{x}\pm s$).

State	Group	Number of cases	4 h	8 h	12 h	24 h	48 h
Resting state	A	36	3.3 ± 0.8	3.4 ± 1.0	3.5 ± 0.7	3.4 ± 0.6	3.2 ± 0.6
	B	35	3.5 ± 0.7	3.4 ± 0.9	3.6 ± 1.0	3.2 ± 0.5	3.3 ± 0.7
	*χ* ^2^		1.578	0.657	0.743	0.476	0.357
	*P*		0.541	0.384	0.681	0.721	0.639

Active state	A	36	3.6 ± 0.6	3.7 ± 0.7	3.8 ± 1.1	3.7 ± 0.8	3.6 ± 0.9
	B	35	3.7 ± 0.4	3.8 ± 0.6	3.9 ± 0.8	3.5 ± 0.6	3.6 ± 0.6
	*χ* ^2^		0.364	0.258	0.697	0.529	0.391
	*P*		0.768	0.539	0.397	0.587	0.648

## Data Availability

All data generated or analysed during this study are included in this published article.
